The article "Health Information Prediction System of Infant Sports Based on Deep Learning Network" was retracted in 2023. Reasons: suspected computer-generated content; unreliable results or conclusions; lack of ethics approval or compliance; missing or withdrawn patient consent.

# Health Information Prediction System of Infant Sports Based on Deep Learning Network

**DOI:** 10.1155/2022/4438251

**Published:** 2022-07-31

**Authors:** Jie Qi, Jun Zhang

**Affiliations:** College of Physical Education, Shanghai Normal University, Shanghai 200234, China

## Abstract

The sensed data from infant sports and training programs are useful in analyzing their health conditions and forecasting any disorders or abnormalities. The sensed information is processed for providing errorless predictions for infant diseases/disorders, coupled with artificial intelligence and sophisticated healthcare technologies. The problem of noncongruent sensed data impacting the forecast occurs due to errors between consecutive training iterations. This problem is addressed using the deep learning (PEST-DL) proposed perceptible error segregation technique. The training process is halted between two consecutive iterations generating errors until a similarity verification based on infant history is performed. The similarity output determines the errors due to mismatching data observations, and therefore, the data augmentation is performed. The first perceptible error is mitigated by training the learning paradigm with all possible infant history data in the learning process. This prevents prediction lag and data omissions due to discrete availability. The learning is trained from the identified error with the precise detected disorder/abnormality data previously detected. Therefore, the first and consecutive training data segregate error instances from the actual training iterations. This improves the prediction accuracy and precision with controlled error and time complexity.

## 1. Background

Sports that underage children play are known as infant sports. Infants' sports are mostly indoor sports that contain various activities to play. Infant sports include reading, clapping, sitting, rolling, walking, crawling, bubble blowing, singing, and playing around the grounds [1]. Data analysis is a process that discovers information and data for the process such as decision-making, detection, and identification process. The infant sports data analysis identifies the information related to the analysis process and produces an optimal set of data for other classification processes [2]. The data analysis process collects information and data necessary for further detection and analysis in sports applications. The bivariate Poisson model is used in the infant sports data analysis to find out the actual details about sports activities and provide needed data for the analysis [3]. The bivariate model first predicts and detects the important details among the information and produces a feasible set of data for the sports data analysis process. The big data analytics method is widely used in infant sports data analysis is the process that finds out the details among the huge amount of data and reduces the latency rate in the identification process. The big data analytics method improves the feasibility and efficiency rate of the infant sports data analysis is the process in sports management systems [4, 5].

The prediction process is a most complicated task in various fields and applications that need to provide an appropriate set of data for further analysis. Sports data is a collection of relevant information and data that provide optimal details for various sports events [6]. Sports data contains details such as the infant's name, age, gender, height, weight, allergies, rashes, activities, and skills collected by performing a certain function. The health prediction of an infant is a crucial task that requires an accurate set of information for the prediction process [7]. Cold, fever, cough, vomiting, and diarrhea are infants' most common health issues, which are needed to predict. The infant health prediction process improves the health condition of infants by increasing the accuracy rate in the prediction process [8]. The gestational age (GA) prediction process is an important health prediction method for the infant that predicts accurate details about the health condition. GA also provides solutions to cure the health conditions of infants that reduce their critical condition of infants [9]. The reduction of infant weight is also a cause of sickness identified by using sports data. Health prediction of infants performs a feature extraction method that finds out the important features of infants and produces a related set of data for the prediction process [10].

The machine learning (ML) technique is widely used in various fields and applications for prediction, detection, recognition, and identification. The ML technique improves the overall accuracy rate in the detection and prediction process and improves the system efficiency [11]. The ML technique is also used in the infant health prediction process by using sports data. The ML technique uses effective classifiers to determine the actual cause of an infant's health problems [12]. Sports data is compared with newly identified data and produced into a feasible set for further analysis. The *k*-nearest neighbor (KNN) algorithm is used in the infant health prediction process that identifies the health condition with a certain set of features and patterns [13]. KNN identifies the important features among the information by performing the classification process. The classification process classifies the data and produces actual information for the prediction process [14]. The support vector machine (SVM) approach is used in the health prediction process that performs regression and classification processes to determine the actual detail of health conditions. Sports data is commonly used in the SVM prediction process, which reduces the latency rate in the data analysis process. A decision tree algorithm is also used to improve the accuracy rate prediction process [15, 16].

The remainder of the research is arranged as follows. Introduction and related work are discussed in Section 1 and Section 2 of this paper, respectively. In Section 3, the PEST-DL system has been suggested. In Section 4, the experimental results have been implemented, and Section 5 concludes the study report.

## 2. Related Works

Wu [17] introduced a human health characteristic of the sports management model using a biometric monitoring system. The proposed model analyzes users' health conditions and gets information from a monitoring system. Body mass index (BMI) rate is identified by the details produced by a biometric monitoring system. The proposed management model improves the effectiveness and efficiency of the management process in a sports environment.

Han and Kim [18] proposed a new overweight and obesity prediction model for children in healthcare centers. A logistic regression algorithm is used to analyze health-related information in the data analysis process. Multidimensional data and features are identified from the healthcare system used for the prediction model. Data such as height, weight, index, and person patterns are collected and stored in the database for further analysis. The proposed model increases the accuracy rate of the prediction model in healthcare systems.

Hamoen et al. [19] introduced a multivariable diagnostic prediction model for high blood pressure in children. The proposed prediction provides accurate details for the diagnosis process that improves the services for the patients. A high blood pressure rate is identified based on certain features and details. Features such as children's height, weight, blood group, parent's health report, and disease are found in the prediction model. The proposed prediction model improves the system's effectiveness by increasing the accuracy rate in the prediction process.

Ruiz et al. [20] proposed a cardiac-intensive-care warning index (C-WIN) system for infants. The Bayesian model is used in C-WIN to determine the problems and events in infants. Routinely collected information is used to get the necessary details for the prediction process. The proposed method is mostly used for predicting congenital heart disease in infants during the incubation process. The proposed prediction method improves the feasibility and performance of infant healthcare systems.

Engan et al. [21] introduced a new physical activity prediction model to find extremely preterm-born children. Preterm-born children are identified based on body mass index (BMI) and extremely low birth weight (ELBW). Sports data is used here to analyze children's physical activities and produce a feasible set of data for the further analysis process. Sports data store details such as low endurance, low energy level, and low proficiency. The proposed physical activity prediction model increases the accuracy rate in the prediction process.

Yun and Edginton [22] proposed a new plasma prediction model for human health risk assessment in children. The proposed prediction model predicts the fraction unbound in plasma for children and produces a proper set of data for the prediction process. A computational tool is used here to fetch the actual details about children's health conditions and plasma features. Experimental results show that the proposed prediction model improves the feasibility and effectiveness of healthcare systems.

León et al. [23] introduced the late-onset sepsis (LOS) prediction method for premature infants using a machine learning approach. The graph analysis process is used here to analyze the information needed for the prediction process. The graph analysis process identifies heart rate visibility (HRV) data and produces an optimal set of data for the LOS prediction process. The proposed prediction model improves the overall performance and efficiency of the system.

Hong et al. [24] proposed a graph-based diffusion MRI data prediction model using a convolutional neural network (CNN) algorithm for infants. Details such as wave-vector domain and sampling information are stored in MRI data. Graph CNN is used here to identify the nonlinear mapping details of MRI data and find out the exact cause of missing diffusion data. The proposed prediction model improves the accuracy rate in the prediction process and increases the system's performance.

Joshi et al. [25] introduced a neonatal sepsis prediction method for infants using heart rate variability (HRV) data. The naïve Bayes algorithm is used in the proposed method to identify the HRV features in infants. Electrocardiogram (ECG) device is used here to capture the activities and conditions of infants that produce an optimal set of data for the prediction process. The proposed method reduces the latency rate in the computation process, which improves the system's efficiency.

Li et al. [26] proposed a transfer learning approach for child activity recognition. Adult-domain data is used here to find out users' activities via accelerometer. Accelerometer capture details such as sitting, walking, running, skipping, and roping users' activities. The classification process is performed in the proposed method to identify the exact details of the child's activities. The proposed method improves the overall accuracy rate in the recognition process.

Lee-Cultura et al. [27] introduced a motion-based learning technology (MBLT) for children's play recognition. A multimodal mixed method is used in MBLT to find out the behaviors and activities of children. The proposed method is mainly used to find out children's learning experiences and produce an optimal dataset for further analysis. Compared with other methods, the proposed recognition method increases the feasibility and effectiveness of the system.

Lan et al. [28] proposed an augmented intercommunication framework (AICF) for identifying sports students' activities. A behavior recognition algorithm is used in AICF that finds out the accurate behavior of students and produces a proper set of data for the recognition process. The proposed method is used to identify students' mental state and condition. The proposed AICF enhances the system's effectiveness, scalability, and performance by improving the accuracy rate in the prediction process.

Chu et al. [29] introduced a sports-related concussion (SRC) recovery prediction method using a machine learning (ML) approach. The proposed prediction method finds out the recovery timing of students by analyzing the injuries. The ML approach is used here to increase the accuracy rate in the prediction process and reduce the latency rate in the computation process. The recovery timing of injuries is calculated and submitted to the management system that provides necessary services for the students. The proposed method reduces the complexity rate in the computation process.

## 3. The Perceptible Error Segregation Technique Using Deep Learning

The proposed objective of this health condition analysis model of infant sports is designed to improve the forecasting of any disorders or abnormalities based on infant history and coupled with sophisticated healthcare technologies. Artificial intelligence sensed data from the wearable and monitoring sensors. In an infant sports health analysis scenario, the sensor devices are used to gather information from the infant, which is forecasted through healthcare systems. These infant data analyses are processed using the sensors for better prediction and variations in diagnosed infant data. The sensor devices gather information in different time intervals to save and update accumulated sensed data from the infant sports and training instance.  Figure 1 portrays the proposed technique and its process.

The proposed technique correctly analyzes grasping and understanding characteristics of the children and the conventional laws of mental and physical development of infants at this stage and developing the targeted infant sports and training are conducted to the growth and physical development of the infant. The first step is to monitor the health condition of children in sports/training in real-time and augment the intelligence of infants' sports/training. A set of sensed data from the children is used to analyze health conditions based on the infant's physical fitness in sports/training. The second step is the detection of any disorders or abnormalities and then any variations in behaviors and nature of mental activities. Artificial intelligence and sophisticated healthcare technologies sensed data from infants providing errorless predictions for children's disorders/diseases. In this process, the problem is addressed due to noncongruent sensed information impacting the forecast at the time of error between sequential training iterations. The main objective is to monitor and analyze sensed data that improve infant sports' prediction accuracy and precision based on deep learning. In the proposed PEST method, the exactness of physical condition and children's growth is analyzed using the deep learning process. The proposed technique is to halt the training process between two consecutive training iterations causing errors until similarity verification based on the previous children's history based on pursuing error reduces the time complexity. The input sensed data are monitored through wearable sensor devices, and children's information can be compared with that all possible previous infant history data in the data healthcare system.

Through sports or training, infant motion and physical condition monitoring are based on sensing data. This is used for diagnosing the healthcare data analysis through infant history In_*H*_ and data (sensed) *S* through wearable and monitoring sensor devices *s* at different time intervals  *T*. Children's healthcare organizations maintain the sensed data processing and their health condition analysis based on forecasting any abnormalities or disorders. The proposed PEST is used to address errors between two consecutive training iterations. The wearable and monitoring sensor is controlled by the healthcare, where smart sports and training for the infants through prediction are made. The prediction of forecast occurs in the infant through monitoring sensors is pursued using the additional sports and training to the infant  *s*_*d*_. The sensed data can be either health condition, sports, training, growth, physical development, mentality, maturity, behaviors, etc. The sensed input data *s*_*d*_ and infant sports and training programs are performed. The deep learning network analyzes the infant's physical condition based on research on a health information prediction system to improve forecasting and detection. Therefore, PEST is coupled into two consecutive iterations: artificial intelligence and sophisticated healthcare technologies.

### 3.1. Consecutive Training Process

The utilization of wearable and monitoring sensor devices is in charge of gathering infant health condition data from the infant's body. The gathered data (sensed) can be of any type based on maturity, nature of mental activities, sports and training, etc. In a data sensing instance, the infant's history In_*H*_ is computed as follows:

(1) $$\begin{array}{c} \left.\begin{array}{c} {\text{In}}_{H}=\frac{\left({s_{d}}_{\max}-{s_{d}}_{\min}\right)}{s_{d}}\\ T=\frac{1}{\sqrt{2\pi }}\left[\frac{\left(\left({s_{d}}_{\min}/{s_{d}}_{\max}\right)-\left(S/s_{d}\right)\right)}{2\left({\text{In}}_{H}-\text{in}\right)}\right] \end{array}\right\}, \end{array}$$

where the variable in is the active infant sensed data gathered and  *S* ∈ *s*_*d*_, and *s*_*d*__max_ and *s*_*d*__min_ are the minimum and maximum wearable and monitoring sensors gathered data sensed at different time intervals. In this previous infant history analysis, the similarity verification is performed between sensed data and pursued health condition analysis. Therefore, *T* and In_*H*_ are used to represent the prediction system at various instances with all possible infant history data. The prediction in the different intervals is estimated as the number of infant history data (sensed) and current forecast occurs observed at different *s*_*d*_ instances. There are some errors due to mismatching data observations to physical condition analysis of  *S*. Hence, this problem results in data augmentation at any interval, for which the infant sensed data is estimated as follows:

(2a) $$\begin{array}{c} S\left({\text{In}}_{H}\right)=\frac{C^{2}}{{\left(\left({s_{d}}_{\min}/{s_{d}}_{\max}\right)-C^{2}\right)}^{2}}. \end{array}$$

Such that

(2b) $$\begin{array}{c} V=\frac{1}{s_{d}}\sqrt{\frac{1}{S-1}\overset{s_{d}}{\underset{T=1}{\sum }}{\left(\frac{{\text{In}}_{H}-\text{in}}{{\text{In}}_{H}}\right)}^{2}}. \end{array}$$

Equations (2a) and (2b) denote the consecutive training iteration based on the sensed data ofIn_*H*_pursuing the prediction which relies on the maximum correlation*C*and the variations in health condition *V*, where *V* is a maximum variation whereas *C* is the medical data correlation at different time instances, for which the errorless prediction of *s*_*s*_ for infant disease/disorders is needed. Based on *s*_*d*_ and  *S*(In_*H*_), the consecutive infant sports and training iteration of data observations is given as in the following equation:

(3) $$\begin{array}{c} T\left[s_{d},S\left({\text{In}}_{H}\right)\right]=\sqrt{{\left[\frac{S\left({\text{In}}_{H}\right)}{s_{d}}\right]}_{1}^{2}+{\left[\frac{S\left({\text{In}}_{H}\right)}{s_{d}}\right]}_{2}^{2}+\cdots +{\left[\left(1-\frac{\text{in}}{s_{d}}\right)C\right]}_{S}^{2},\;\;S\in s_{d}}. \end{array}$$

Equation (3) computes the consecutive training iteration in the different time intervals for an instance until the forecast occurs due to an error in sensing data from the infant body based on healthcare systems. The similarity verification, diagnosis data, and error segregation process are performed using deep learning.  Figure 2 presents the training and iteration required for data analysis.

The input  *S* = *S*_*d*_ + *S*_*d*__max_ is classified at the initial stage for further segregation. Based on *T* and  *S*(*In*_*H*_)∀ *V*, the  *T*[*S*_*d*_, *S*(*In*_*H*_)] is accumulated.  *In*_*H*_ is used for validation based on training. The  *S* ∉ *In*_*H*_ (or)  *S* ≠ {1, 2, ⋯, *T*} is used for training the learning paradigm. Therefore, the error classification is eased by identifying the diagnosed (from  *In*_*H*_) data (refer to Figure 2). The sensed data based on physical information correlated and examined using the learning process. In this infant health information prediction, the gathered input felt data is to be matched into previous infant history that outputs in data augmentation based on the accurate and exact time interval to augment the precision accuracy of children's health data prediction system. Instead, the data augmentation is verified with the healthcare data through deep learning. Therefore, data augmentation of the similarity output determines the errors due to mismatched during data observation through deep learning, like the diagnosis of data used for *S* computation. The solution of the deep learning is to identify prediction, healthcare data, and process error segregation, which relies on In_*H*_ assessment and in based sequence. Initially, the learning method is to maintain the errorless prediction for infant disease/disorder if  *T* is observed at any instance. The similarity verification succeeding (1 − (in/In_*H*_))*C* at the infant history is the precise output for error segregation. In this manner, the data observations due to mismatched physical data employed with all possible infant history data and noncongruent sensed data impacting the forecasted healthcare data. Therefore, the two consecutive iterations generate errors of *s*_*d*_. In any instance, *i* and *j* are forecast of the sensed data through deep learning. For *T* assessment, the sequence of iterations is modeled as per the equation:

(4) $$\begin{array}{c} \left.\begin{array}{c} \left.\begin{array}{c} i=s_{d}\\ j=0 \end{array}\right\},\text{the initiating iteration}\\ \left.\begin{array}{c} i=S\left({\text{In}}_{H}\right)\\ j=\frac{V}{C} \end{array}\right\},\text{the consecutive iteration} \end{array}\right\}, \end{array}$$

where

(5) $$\begin{array}{c} \left.\begin{array}{c} i+j=s_{d}\text{ is the input for first iteration}\\ S\left({\text{In}}_{H}\right)+\frac{V}{C}\text{ is the input for consecutive iteration} \end{array}\right\}. \end{array}$$

The similarity verification assessment from the two consecutive training iterations is based on matching with the infant history data. In this *s*_*d*_, if the similarity is observed at any instance, prediction is provided, where in PEST-DL, the two consecutive iterations of *i* + *j* = *S*(In_*H*_) + *V*/*C* are observed for identifying error segregation from the actual training instances. The error identification process from the first and consecutive learning iterations is illustrated using Figure 3.

The  *In*_*H*_ ∈ *S* and ∉*S* are classified in Figure 2, for which the hidden layer mapping ∀*i*  to  (*i* + *n*) and  *j* to (*j* − *n*) is performed. Based on the classifications using Equation (5) for  *S*(*In*_*H*_) and  *V*, the  *S*{*T*[*S*_*d*_, *S*(*In*_*H*_)]} is identified. The  *S*_*d*__max_∀ *V* in distinguishable iterations,  *i* to  (*i* + *m*), i.e.,  (∑*i* + *n*) , generates matching data. This is used for training and learning improvements. Contrarily, the  *j* to  (*j* + *n*) generates  *D*_*o*_ in the first classification pursued by (*P*_*l*_ − *D*_*o*_)  in successive iterations. These two classifications are generated as abnormal/error-causing outputs (refer to Figure 3). The joint first and consecutive training data are used for segregating errors from the available training iteration *S*, and its related activities are analyzed by the PEST method. They are discussed as per the following equation.

(6) $$\begin{array}{c} \left.\begin{array}{c} S\left\{T\left[s_{d},S\left({\text{In}}_{H}\right)\right]\right\}=iE^{L}-js_{d}-E^{L}s_{d}A^{D}\\ \text{such that}\\ \begin{array}{c} i\left(E^{L}\left|s_{d}\right.\right)=e\left(s_{d}+A^{D}E^{L}\right)\\ j\left(s_{d}\left|A^{D}\right.\right)=e\left(i-A^{D}E^{L}\right) \end{array} \end{array}\right\}. \end{array}$$

In Equation (6), the variable *E*^*L*^ is the errorless prediction of the precision accuracy and *A*^*D*^ is the data augmentation factor observed by similarity verification based on *s*_*d*_ and  *i*,  *j* with  *E*^*L*^. Based on the condition, *i*(*E*^*L*^|*s*_*d*_) and *j*(*s*_*d*_|*A*^*D*^) are the data observation that is used for satisfying the condition  *S*{*T*[*s*_*d*_, *S*(In_*H*_)]}. As discussed in Equation (5), with all possible infant data, either achieve *i*(*E*^*L*^|*s*_*d*_) or *j*(*s*_*d*_|*A*^*D*^) for all the consecutive training iterations based [*s*_*d*_ ± *A*^*D*^*E*^*L*^] and  [*i* ± *A*^*D*^*E*^*L*^]. The data augmentation and deep learning of the infant physical data observation based on the above representation analyzed for error occurrence *i* ± *j* are to satisfy the above data observation. From the above representation, the consecutive training instances based on *i*(*E*^*L*^|*s*_*d*_) and  *j*(*s*_*d*_|*A*^*D*^) and the assessment of *A*^*D*^*E*^*L*^ and *S*(In_*H*_) outputs in mismatching data observations generate the error of *S*{*T*[*s*_*d*_, *S*(In_*H*_)]} as its least possible error prediction. In this process, the deep learning for infant health information is the prediction system follows  *i*, *j* and  *T*[*s*_*d*_, *S*(In_*H*_)], followed by the data augmentation based on similarity verification through in and *A*^*D*^.

As different infant sports and training, precision accuracy of physical information prediction system of data augmentation and observation is analyzed. However, to control the prediction errors reducing the time complexity during training instances is mandatory. The proposed technique provides better data observation with all infant history data. Let {1, 2, ⋯, *E*^*L*^} ∈ *e* denote a set of infant sports/training based on input data analyzed in different intervals [*T* ∈ (*P*_*l*_ − *D*_*O*_)], where *P*_*l*_ and *D*_*O*_ are the prediction lag and data omissions due to discrete data availability, respectively. From different instances, the further processing  *s*_*d*_ and the prediction system *p*_*s*_ must be less under detected disorder/abnormality data observed that is computed as follows:

(7) $$\begin{array}{c} \forall \left(P_{l}-D_{O}\right),\text{argmin }\overset{p_{s}}{\underset{T=1}{\sum }}\frac{\left(s_{d}-E^{L}\right)}{e},\;\;T\in \left[P_{l}+1,D_{O}\right]. \end{array}$$

Such that

(8) $$\begin{array}{c} \text{argmin }\overset{E^{L}}{\underset{t=1}{\sum }}P_{l}*p_{s}\forall \left\{1,2,\cdots ,E^{L}\right\}\in e,\;\;D_{O}\leq T\leq P_{l}, \end{array}$$

where the variable *E*^*L*^ denotes the errorless prediction based on medical data analysis and (*s*_*d*_ − *E*^*L*^) in the previous abnormality data detection in any  *T* ∈ [*P*_*l*_ + 1, *D*_*O*_]. This consecutive training iteration reduces the errors in a different instance, reducing the prediction lag and data omissions due to discrete availability.

The above problem is addressed using the previous data observation and new infant sensed data of the health information prediction system through the deep learning process. Therefore, there are few constraints based on *D*_*O*_ and *c*_*R*_ that is evaluated as ∀*E*^*L*^ ∈ *p*_*R*_ in  [*P*_*l*_, *D*_*O*_], if (*E*^*L*^ + 1) is true in  *D* ∈ [*P*_*l*_ + 1, *D*_*O*_], and then, (*E*^*L*^ + 1) experience a data detected previously in different time instances of  (*T* + *P*_*l*_ + 1 ), where  *T* represents the data omissions and ∀*E*^*L*^ ∈ *s*_*d*_ in  *P*_*l*_, if *T* = *D*_*O*_/*T* > *D*_*O*_, and then, Δ = (*s*_*d*_ − *p*_*s*_) is maximum in reducing the error and*p*_*s*_/*s*_*d*_⟶0.

In this consecutive training iteration instance, the variable  *e* represents the prediction error. The first condition determines the errorless prediction output (*P*_*l*_ − *D*_*O*_), where the second condition outputs in the new sensed data observation can be similar to all possible infant history data  *E*^*L*^, i.e.,  (*E*^*L*^ + 1), if there is a joint first with any instance  *T* ∈ [*P*_*l*_ + 1, *D*_*O*_] of  *E*^*L*^. This maximizes the perceptible error between  *E*^*L*^ and  (*E*^*L*^ + 1). From the discrete availability, the data omission and prediction lag are processed as  [*P*_*l*_ − *D*_*O*_] different interval and also checking whether if it is suspended with the successive  *p*_*s*_ requires their health conditions and forecasting any abnormalities/disease based on the condition argmin∑_*T*=1_^*p*_*s*_^*P*_*l*_∗*p*_*s*_∀ [*P*_*l*_ − *D*_*O*_] is achieved.

This error segregation and abnormality detection of ∑_*T*=1_^*p*_*s*_^*P*_*l*_∗*p*_*s*_∀ [*P*_*l*_ − *D*_*O*_] is valid until the similarity verification fails. Instead, forecasting varies both joint and consecutive training data instances until it is idle either for continuous or discreteness. The prediction lag and data omission are analyzed based on discrete data availability that is aided for data augmentation. Then, the detection process is performed based on the variations in the medical data. The identification of  *e* is addressed due to changes in infant sports/training from discrete availability instances or vice versa. Therefore, there is a maximum possible forecast occurrence due to errors that are misguided as  *e*; in the above similarity verification and actual training instance, the data augmentation improves the chances of errors to reduce the time complexity.

## 4. Performance Assessment

The data input for injury data prediction is used in the performance assessment section. This is used for assessing the health of children between 0 and 14years of age group [30]. For more precise information handling, 605 inputs out of 2461 entries are alone considered for analysis. The dataset representation with the correlation to the proposed technique is illustrated in Figure 4.

The input dataset is exploited as represented above, wherein the lower- and upper-level variations are identified for  *D*_*o*_. Contrarily, the absolute data value for variation 2 (as shown above) is estimated as  *p*_*l*_ − *D*_*o*_. The first observation for training is identified from the first entry until the same  (*In*_*H*_) is not observed. Based on variations 1 and 2, the learning is instigated from the data estimated. Based on this information, the analysis for  *S*_*d*_ and *s*_*d*_max__ observed is presented in Figure 5. In this, analysis for  *i* and  *j* is also presented.

In Figure 4, the  *S*_*d*_, *S*_*d*_max__ from the input data is identified from different iterations for  “*i*” and “*j*” as estimated in Equation (4). This estimation generates consistent (high-level) outputs for varying iterations. The input contains a variation from 12.3 to 684.062, from which the predicted output using the proposed technique is alone analyzed. Based on this information, the variation, i.e., *D*_*o*_, and variation 2, i.e.,  (*P*_*l*_ − *D*_*o*_), for lower and upper levels under “*i*” and “*j*” are tabulated in Table 1.

In the above table, variations 1 and variation 2 are analyzed under different iterations for “*i*” and “*j*”. It is seen that the proposed technique reduces the error for  *D*_*o*_ and (*P*_*l*_ − *D*_*o*_) in “*j*” greatly, compared to “*i*”. This is due to the joint training of  *S*_*d*_, *S*_*d*_max__ and  *S*(*In*_*H*_) from different iterations. Therefore, as the iteration increases,  (*i* + 1) and *v*/*c*  are classified for preventing variation that ∉*S*(*In*_*H*_) is observed. In Figure 6, the  *T* accuracy over the varying iterations for “*i*” and “*j*” (cumulatively) under lower- and upper-level values is presented.

As the iteration increases, the joint combination of*S*_*d*_, *S*_*d*__max_, and *S*(*In*_*H*_)achieves high accuracy for “*j*” than “*i*”. The lower- and upper-level data are analyzed for detecting accuracy under distinct  *D*_*o*_ and  (*P*_*l*_ − *D*_*o*_). The learning process segregates errors for improving the training rate in “*i*” such that  *S* = *S*_*d*_ + *S*_*d*__max_ is alone utilized if variation 1 (or) variation 2 (or) both are for preventing error invalidation. Therefore, the detection accuracy is stabilized for the training process (refer to Figure 6). In the comparative analysis, the methods TL-CAR [26], MLRA+DT [18], and AICF [28] are considered for validating accuracy, precision, error, and time complexity.

### 4.1. Accuracy

In Figure 7, the health information prediction system of infant sports/training is useful in analyzing their health conditions and forecasting any diseases or abnormalities by providing artificial intelligence. Sophisticated healthcare technologies based on the sensed information improve the precision accuracy through deep learning which does not provide consecutive training iterations depending on the similarity verification based on infant history at different intervals. The variations in health conditions with all possible infant history and real-time physical information from the first step outputs in similarity enhance the precision and prediction accuracy for the data observations wherein the sensed data and healthcare data based on the infant sports and training data can be extracted. This impact is addressed using deep learning, and data augmentation can be analyzed to satisfy successive errorless predictions based on the sensor data depending on the mismatched data, preventing errors. Therefore, the diagnosed data based on the variations in children's health conditions are detected, preventing high accuracy due to the new sensed data in identifying the error.

### 4.2. Precision

The data augmentation provides the similarity output that determines the errors based on infant diseases/disorders detected for the health information prediction as the first step data observation based on the nature of mental activities. Physical information is deployed for error segregation based on the constraints. Noncongruent sensed data is represented in Figure 8. This proposed technique satisfies high prediction accuracy by computing the prediction lag and data omission instances. In this analysis, the previous infant history data is processed until the new data is sensed based on healthcare data at different intervals to prevent data omission. The previously detected abnormality mitigation based on the similarity verification is computed until sensed data impacting during forecast occurs. This error is accounted for using suspension based on the third iteration, and data augmentation can be analyzed for satisfying successive errorless predictions. Therefore, the correlation and diagnosis based on medical data of infants are maximized, and variations due to physical changes in the infant body provide consecutive training which is high precision with all possible infant history data.

### 4.3. Error

The infant's physical condition is based on forecasting disorders or abnormalities detected based on artificial intelligence, and sophisticated healthcare technologies depend on the infant's sensed information in different time intervals as represented in Figure 9. In this prediction system on infant sports, the abnormal activity detection is based on different instances, such that *i* + *j* = *S*(In_*H*_) + *V*/*C* the forecast occurs due to errors between consecutive training iterations. The sensed data analysis is based on the discrete availability of input data observations. The disease and abnormalities are detected in the forecasted monitoring sensors based on similarity verification and mismatching. The different training iterations with the precisely detected abnormalities are analyzed based on the data augmentation. In this proposed technique, the perceptible error is mitigated by training abnormal activity detection infants through a deep learning process based on two conditions analyzed for further estimation of error which is considered for providing additional training for the abnormality detected children. Therefore, the prediction error is less compared to the other factors in infant health condition prediction based on consecutive training instances, and the error is detected.

### 4.4. Time Complexity

In this proposed infant physical condition monitoring through sensors, disorders/abnormalities are detected at any time interval based on time complexity. It causes errors in data observation depending on the correlation process based on two consecutive iterations that provide similarity verification through deep learning. The assessment of disease or disorder detection in the children based on the infant history mismatching condition  *D* ∈ [*P*_*l*_ + 1, *D*_*O*_] and then (*E*^*L*^ + 1) is computed using data augmentation for the first error occurrence for *D*_*O*_ ≤ *T* ≤ *P*_*l*_ which impacts the consecutive training iterations of abnormal activities detected based on monitoring infant health information which can be analyzed for both conditions using deep learning. Based on the infant's history, similarity verification is processed based on present health condition with history in any time interval, preventing time complexity. The proposed disease or disorder detection of children through deep learning depends on errorless prediction. The identified error instance from the actual training iterations achieves less time complexity, as presented in Figure 10.  Table 2 and Table 3 present the comparative analysis result for varying  *S* intervals and mismatching rates.

## 5. Conclusion

This article presents a perceptible error segregation technique for infant/children health data analysis based on prediction. The proposed technique is supported by a deep learning paradigm for identifying errors in training iterations. The sensed data is differentiated under initial and consecutive variation detection sequences. This sequence identifies the similarity between the medial data history and mismatching instances. The training is prevented from handling error data for continuous iteration observations. Therefore, the new data augmentations are initiated from the similar maximum data and the error-causing instance. This is performed from the consecutive training process to reduce time complexity. Based on the error from the consecutive learning process, the disorder and abnormality are validated through different segregation instances, improving precision. For the varying  *S* interval, the proposed technique achieves 9.24% high accuracy, 7.67% high precision, 8.22% less error, and 9.7% less time complexity.

## Figures and Tables

**Figure 1:** Proposed PEST-DL.

**Figure 2:** Training and iteration required data analysis.

**Figure 3:** Error identification from first and consecutive learning iterations.

**Figure 4:** Dataset representation.

**Figure 5:** Upper and lower values for *S*_*d*_ and *s*_*d*_max__ under varying iterations.

**Figure 6:** *T* accuracy over the varying iterations.

**Figure 7:** Accuracy analysis.

**Figure 8:** Precision analysis.

**Figure 9:** Error analysis.

**Figure 10:** Time complexity analysis.

**Table 1:** Variations 1 and 2 for varying iterations.

Iteration	Variation 1		Variation 2	
	*i*	*j*	*i*	*j*
100	0.353	0.399	0.0424	0.02738
200	0.41	0.631	0.3598	0.2347
300	0.322	0.512	0.3158	0.01985
400	0.312	0.451	0.02897	0.0158
500	0.256	0.652	0.02658	0.00986
600	0.24	0.841	0.01708	0.00639

**Table 2:** Comparative analysis result for varying *S* interval.

Metrics	TL-CAR	MLRA+DT	AICF	PEST-DL	Inference
Accuracy (%)	78.85	85.61	89.77	93.986	9.24% high
Precision	0.817	0.864	0.917	0.9427	7.67% high
Error	0.21	0.152	0.129	0.0815	8.22% less
Time (s)	0.259	0.192	0.132	0.0814	9.7% less

**Table 3:** Comparative analysis result for varying mismatching rate.

Metrics	TL-CAR	MLRA+DT	AICF	PEST-DL	Inference
Accuracy (%)	73.16	79.73	82.64	86.06	7.55% high
Precision	0.774	0.801	0.839	0.8913	8.66% high
Error	0.203	0.159	0.117	0.0767	8.3% less
Time (s)	0.249	0.192	0.126	0.0818	9.45% less

## Data Availability

The data that support the findings of this study are available from the corresponding author upon reasonable request.
